The article "Low fruit and vegetable intake is associated with depression among Korean adults in data from the 2014 Korea National Health and Nutrition Examination Survey" was published in 2019. Journal: J Health Popul Nutr.

# Low fruit and vegetable intake is associated with depression among Korean adults in data from the 2014 Korea National Health and Nutrition Examination Survey

**DOI:** 10.1186/s41043-019-0204-2

**Published:** 2019-12-03

**Authors:** Se-young Ju, Yoo Kyoung Park

**Affiliations:** 1 Dept. of Food Bioscience, Konkuk University, Chungju, 27478 South Korea; 2 Dept. of Medical Nutrition, Graduate School of East-West Medical Science, Kyung Hee University, Yongin, 17104 South Korea; 3 Institute of Medical Nutrition, Kyung Hee University, Seoul, 02447 South Korea

**Keywords:** Fruits and vegetables, Depression, National Health and Nutrition Examination Survey, Odds ratio

## Abstract

**Background:**

Depression is a major mental disorder worldwide. The prevalence of depression among Korean adults was estimated to be 5.6% in 2006 and 6.7% in 2011, and that increased to 10.3% in 2013. Using national data, the present study investigated the association between vegetable and fruit intake and the prevalence of depression among Korean adults.

**Methods:**

This analysis used data from 4349 subjects aged 19 years and older who participated in the Korea National Health and Nutrition Examination Survey (KNHANES, 2014). Depression was assessed using the self-reported Patient Health Questionnaire (PHQ)-9. Food and nutrient intake was assessed using the 24-h recall method. Individual food intake was categorized into 18 food groups. The statistical analyses in this study were performed by adopting stratification, clustering, and sample weight variables using SPSS Ver. 23.0. Cronbach’s α was used to determine the internal consistency of the PHQ-9 items. Logistic regression analysis was used to estimate the odds ratios of depression adjusted for several confounders.

**Results:**

The depression rate of all subjects was between 8.7 and 4.7% and decreased as vegetable and fruit intake increased. With regard to sex, the depression rate decreased from 6.4 to 2.5% in males and from 11.4 to 6.6% in females as vegetable and fruit intake increased. Thus, the results of this study reveal an inverse association between vegetable and fruit intake and depression. The odds ratios show that vegetable and fruit intake was inversely associated with depression with no adjustment. When the data were adjusted for age, energy intake, obesity, smoking, drinking, stress, eating-out frequency, breakfast, and food security, subjects exhibited significantly lower rates of depression with higher vegetable and fruit intakes.

**Conclusions:**

This is the first study to investigate the association between vegetable and fruit consumption and depression in a Korean population. Additional epidemiological studies are needed to find the underlying reasons for that association.

## Introduction

Depression is a major mental disorder worldwide. According to reports from the World Health Organization, the global prevalence of depression is 4.3%, with an incidence of 3.0%, and the condition is one of the leading causes of disability around the world [1, 2]. The prevalence of depression among Korean adults was estimated to be 5.6% in 2006 and 6.7% in 2011, and that increased to 10.3% in 2013 [3]. Depression is a mood disorder that includes feelings of worthlessness, being overwhelmed, and a lack of confidence. It is related to reduced productivity and poor quality of life and can give rise to a higher risk of suicide [4]. The causes of depression have not been clearly identified, but they are known to be related to a variety of biological, genetic, psychological, and environmental factors [5]. In recent years, dietary nutrients have received attention for their potential to prevent and treat chronic diseases, including depression. Several healthy dietary patterns, such as the Mediterranean (high in vegetables, fruits, and olive oil) [6–8], traditional Japanese (rich in fruit, vegetables, green tea, and soy) [9], and traditional (rich in vegetables, fruit, fish, and unprocessed meat) [10, 11] diets, have all been reported to be negatively associated with depressive symptoms. On the other hand, unhealthy dietary patterns, including processed foods such as sweets, fried food, processed meats, refined grains, and high-fat dairy [12], and a Western diet [9, 11, 13] have been reported to be positively associated with the odds of depression. More evidence of an inverse association between fruit and vegetable consumption and depression in a Western population was reported by McMartin et al. [14], Mihrshahi et al. [15], Johnson et al. [16], and Ribeiro et al. [17]. Bishwajit et al. [18] reported that daily intake of fewer than five servings of fruits and vegetables was associated with higher odds of depression in a south Asian population. However, the prevalence of self-reported depression in Bangladesh, India, Nepal, and Sri Lanka averaged more than 35%, which seems to be an overestimation.

Studies of the association between vegetable and fruit intake and depression in the Korean population, whose average intake of fruits and vegetables is relatively high, are lacking, limited to an examination of the relationship between dietary patterns and depression in adolescent girls [19] and Korean adults [20]. Therefore, we used data from the 2014 Korea National Health and Nutrition Examination Survey (KNHANES) to investigate the association between vegetable and fruit intake and the prevalence of depression among Korean adults.

## Methods

### Subjects and general characteristics

We used data from the 2014 KNHANES for 4349 subjects aged 19 years and older. Individuals who did not participate in the health behavior interviews and 24-h dietary recall tests and those who reported eating fewer than 500 kcal or more than 5000 kcal of daily total caloric intake were excluded to minimize biases (Fig. 1). All the KNHANES questionnaires used in this study were approved by the Institutional Review Board of the Korea Centers for Disease Control and Prevention (approval number: 2013-12EXP-03-5C).

**Fig. 1:** Flow chart for the selection of study subjects

The general characteristics of the subjects were analyzed according to sex, age, marital status, residential area, occupational status, educational level, household income, and average family size. Age was classified as follows: 19 to 29, 30 to 49, 50 to 64, 65 to 74, and 75 years and older. Residential areas were classified as “city” and “rural.” The following classifications were also used: household income (low, middle-low, middle-high, and high), educational level (middle school or less, high school or less, and college degree or more), and occupational status (employed and unemployed).

### Depression measures

Subjects with depression were selected based on their answers to the Patient Health Questionnaire (PHQ)-9 part of the health survey in the 2014 KNHANES. The PHQ-9 is a self-rated diagnostic tool for depression listed in the Diagnostic and Statistical Manual of Mental Disorders, Fourth Edition [21–24]. It is a widely used and well-validated measure for monitoring depressive symptoms [25]. Han et al. [24] validated a Korean version of the PHQ-9 that is used in clinical trials and medical research settings to assess depression. Participants were asked, “How often have you been bothered by any of the following symptoms over the previous two weeks?” The PHQ-9 uses nine items to measure the severity of depressive symptoms: little pleasure in activities, feelings of hopelessness or feeling down, sleep disturbances (trouble falling asleep or staying asleep or sleeping too much), feeling tired or having little energy, changes in appetite (poor appetite or overeating), feelings of guilt or worthlessness, trouble concentrating, feeling lethargic or fidgety, and feeling suicidal [26]. Each of the nine items is rated on a four-point scale of 0 (not at all), 1 (several days), 2 (more than half the days), and 3 (every day), and the answers are summed to provide the total PHQ-9 score. Based on previous studies, subjects with PHQ-9 score ≥ 10 (of 27 points) were defined as having depression in this study [23, 24, 26, 27].

### Health behavior measures

The health behaviors assessed in the current study were smoking status (non-smoker, ex-smoker, or current smoker), drinking status (≥ 4 times/week, 2–3 times/week, 1–4 times/month, or < 1 time/month), stress status (very much, somewhat, a little, and rarely), and exercise status (< 1 day/week, 1–2 days/week, 3–4 days/week, and ≥ 5 days/week). Based on body mass index (BMI kilograms/square meter), the weight status was divided into four groups: underweight (< 18.5), normal (18.5–23.0), overweight (23.0–25.0), and obese (≥ 25.0).

### Dietary behavior measures

The number and type of meals consumed (breakfast, lunch, and dinner) and the average frequency per week of eating out (≥ 2 times/day = 14, once per day = 7, 5–6 times/week = 5.5, 3–4 times/week = 3.5, 1–2 times/week = 1.5, 1–3 times/month = 0.32, rarely = 0) were analyzed. Four groups of food security status were identified according to the dietary survey included in the KNHANES data [28]: “food secure” (able to meet essential food and non-food needs for all family members without depletion of assets), “mildly insecure” (minimally adequate food consumption but unable to afford some essential non-food expenditures without depletion of assets), “moderately insecure ” (marginally able to meet minimum food needs because of insufficient money), and “severely insecure” (often not enough food to eat because of insufficient money, has large food consumption gaps).

### Food intake

Food intake was assessed using the 24-h recall method. Based on previous studies [29, 30], individual food intake was categorized into 18 food groups: total food, cereals and grain products, potatoes and starches, legumes and their products, seeds and nuts, sugars and sweets, vegetables, fruits, seaweeds, fish and shellfish, meat, poultry and its products, oils and fats, seasonings, mushrooms, eggs, milk and dairy products, beverages, and other foods. Vegetables were classified into two categories of non-salted or non-starchy vegetables (excluding pickled and salted vegetables, starchy vegetables, and juice) and salted vegetables (including pickles, kimchi, and fermented vegetables). Fruit was categorized as fresh fruit (excluding jams, sweetened fruits, and juices) and sweetened fruit (including jams).

### Statistical analysis

The KNHANES was conducted using a nationally representative estimate of the Korean population based on a multistage, stratified, cluster sampling method. The statistical analyses in this study were performed by adopting stratification, clustering, and sample weight variables using SAS version 9.4 statistical software (SAS Institute, Cary, NC, USA). Cronbach’s α was used to determine the internal consistency of the PHQ-9 items. For general characteristics and health and dietary behaviors according to depression status, the results are reported as frequency and weighted percent from the frequency analysis. Chi-squared testing was used to identify significant differences among categorical variables. For the PHQ-9 items of age, family size, average eating-out frequency per week, average meal frequency per day, BMI, average sleep time, and food and nutrient intake according to depression status, means and standard errors were calculated using the surveymean procedure. Significant differences were verified using an unadjusted *t* test. A generalized linear model was used after adjusting for sex, age, and energy intake with the surveyreg procedure. The correlation between vegetable/fruit intake and depression was determined using a logistic regression analysis with quartile groups (Q1, Q2, Q3, Q4) of non-salted vegetables and fresh fruit intake as the independent variable and depression status (depression, 1; normal, 0) as the dependent variable using the surveylogistic procedure. The amount of non-salted vegetables and fresh fruits eaten was divided into quartiles, and the lowest quartile (smallest consumption of vegetables and fruits) was used as the reference category. The results are presented as odds ratios (ORs) with 95% confidence intervals (CIs). The logistic regression analysis was performed after adjusting for sex, age, energy intake, smoking, drinking, exercise, stress, snacks, breakfast, marital status, eating-out frequency, food security, and household income in stages.

## Results

Table 1 presents the mean and standard error for each item in the PHQ-9 and Cronbach’s α for the internal consistency of the PHQ-9. Cronbach’s α was 0.808, and the total PHQ-9 scores in the depression and non-depression groups were 13.8 and 2.1, respectively. Item 4 (feeling tired or having little energy) was ranked highest among the PHQ-9 items, followed by item 3 (trouble falling or staying asleep or sleeping too much). Item 8 (moving or speaking so slowly that other people have noticed) was the lowest rated.

**Table 1:** Average points and reliability of PHQ-9 items according to the prevalence of depression

Patient Health Questionnaire-9	Non-depression^1^ (*n* = 4050)		Depression^2^ (*n* = 299)		Total (*n* = 4349)	
	Mean	SE	Mean	SE	Mean	SE
1. Little interest or pleasure in doing things	0.3^3^	0.01	1.7	0.1	0.4	0.01
2. Feeling down, depressed, or hopeless	0.2	0.01	1.8	0.1	0.3	0.01
3. Trouble falling or staying asleep or sleeping too much	0.4	0.02	2.2	0.1	0.6	0.02
4. Feeling tired or having little energy	0.6	0.02	2.4	0.1	0.7	0.02
5. Poor appetite or overeating	0.2	0.01	1.5	0.1	0.3	0.01
6. Feeling bad about yourself—or that you are a failure or have let yourself or your family down	0.1	0.01	1.5	0.1	0.2	0.01
7. Trouble concentrating on things, such as reading the newspaper or watching television	0.1	0.01	1.0	0.1	0.1	0.01
8. Moving or speaking so slowly that other people could have noticed. Or the opposite, being so fidgety or restless that you have been moving around a lot more than usual	0.04	0.004	0.8	0.1	0.1	0.01
9. Thoughts that you would be better off dead or of hurting yourself in some way	0.05	0.004	0.9	0.1	0.1	0.01
Total score	2.1	0.04	13.8	0.2	2.8	0.1
Cronbach’s α	0.808					

^1^Total score of PHQ (Patient Health Questionnaire)-9 < 10

^2^Total score of PHQ-9 ≧ 10

^3^Q. 1–9. Score (0: Not at all, 1: Several days, 2: More than half the days, 3: Every day)

The general characteristics of the subjects according to depression are presented in Table 2. The non-depression and depression groups composed 93.5% (*n*, 4050) and 6.5% (*n*, 299) of the total, respectively. The prevalence of depression in females (68.5%) was significantly higher than in males (31.5%) (*P* < 0.0001). People of both sexes aged 30–49 years showed the highest percentage of depression among all age groups (non-depression group, 40.5%; depression group, 31.4%). Regarding the education level, the college or higher group showed the highest depression among all groups (non-depression group, 49.3%; depression group, 40.4%) (*P* = 0.0006). Depression in the unemployed group (55.8%) was significantly higher than in the employed group (44.2%) (*P* < 0.0001). In addition, depression in the low household-income group (34.1%) was significantly higher than in the other income groups (*P* < 0.0001). The average family size in the non-depression and depression groups was 3.2 and 2.8, respectively (*P* = 0.0001). Regarding smoking, nonsmokers showed higher depression (60.9%), followed by ex-smokers (*P* = 0.0115). Drinking < 1/month was associated with the highest depression (50.3%) among all drinking groups (*P* = 0.0097). The stress status responses “feel somewhat” (44.0%) and “feel it very much” (32.3%) had the highest association with depression (*P* < 0.0001). Sleeping hours for the depression group were lower than those for the non-depression group (*P* = 0.007). With respect to weight status associated with depression, the normal group (40.5%) showed the highest depression, followed by the obese, overweight, and underweight groups (*P* = 0.0147). Depression rates by exercise level did not differ significantly between groups. With respect to daily meals, skipping lunch was significantly associated with the depression group compared to the non-depression group (*P* = 0.0080). With respect to food security, the “mildly insecure” group showed the highest depression (49.4%), followed by the “food secure,” “moderately insecure,” and “severely insecure” groups (*P* < 0.0001). With respect to eating-out frequency per week, the averages in the depression group and non-depression group were 3.3 and 4.3 times, respectively (*P =* 0.001).

**Table 2:** General characteristics of subjects according to the presence of depression

	Non-depression (*n* = 4050)		Depression (*n* = 299)		*P* value^2^
	*n*	%^1^	*n*	%	
Total	4050	93.5	299	6.5	-
Sex					
Male	1674	50.3	70	31.5	< 0.0001
Female	2376	49.7	229	68.5	
Age					
19–29 years	423	18.5	40	23.0	0.0059
30–49 years	1388	40.5	77	31.4	
50–64 years	1135	25.6	77	23.0	
65–74 years	722	10.3	63	14.4	
75 years or older	382	5.2	42	8.1	
Average age (mean, SE)	46.1	0.5	46.9	1.3	0.5030^3^
Marital status					
Married	3494	77.9	246	73.2	0.1466
Single	556	22.1	53	26.8	
Education level					
Less than high school graduation	1337	22.5	143	33.5	0.0006
High school graduation	1098	28.1	68	26.1	
College or higher	1612	49.3	88	40.4	
Area					
City	3261	84.1	240	87.4	0.1650
Rural area	789	15.9	59	12.6	
Occupation					
Employed	2364	63.8	114	44.2	<0.0001
Unemployed	1684	36.2	185	55.8	
Household income level					
Low	726	12.6	126	34.1	< 0.0001
Middle-low	1016	25.1	72	25.1	
Middle-high	1186	31.4	51	17.3	
High	1111	30.9	49	23.5	
Family size (mean, SE)	3.2	0.04	2.8	0.1	0.0001^3^
Smoking status					
Current smoker	707	22.8	59	27.5	0.0115
Ex-smoker	784	19.8	40	11.6	
Non-smoker	2517	57.4	196	60.9	
Drinking status					
< 1/month	1927	42.0	170	50.3	0.0097
1–4/month	1248	35.0	72	29.6	
2–3/week	562	16.3	30	10.7	
≧ 4/week	275	6.7	25	9.5	
Stress status					
Feel it very much	97	2.6	85	32.3	< 0.0001
Feel somewhat	698	19.2	127	44.0	
Feel a little	2396	61.4	66	19.0	
Rarely	817	16.8	17	4.7	
Sleeping hours (mean, SE)	6.8	0.02	6.4	0.1	0.007^3^
Exercise					
< 1/week	1910	45.6	167	51.1	0.1695
1–2/week	599	15.6	35	14.4	
3–4/week	594	15.1	29	10.2	
≧ 5/week	947	23.8	68	24.3	
Obese status					
Underweight (BMI < 18.5 kg/m^2^)	161	4.2	26	8.9	0.0147
Normal (18.5 kg/m^2^ ≤ BMI < 23 kg/m^2^)	1660	41.8	123	40.5	
Overweight (23 kg/m^2^ ≤ BMI < 25 kg/m^2^)	954	22.5	60	18.6	
Obese (BMI ≥ 25 kg/m^2^)	1275	31.5	90	32.0	
BMI (mean, SE)	23.7	0.1	23.5	0.3	0.6832^3^
Daily meals (skipped)					
Breakfast	747	23.6	64	29.0	0.0687
Lunch	317	8.9	39	14.8	0.0080
Dinner	248	6.3	22	8.5	0.2240
Food security					
Food secure	2085	52.0	102	34.9	< 0.0001
Mildly insecure	1800	44.4	143	49.4	
Moderately insecure	124	3.0	34	10.8	
Severely insecure	32	0.6	17	5.0	
Frequency of eating-out per week (mean, SE)	4.3	0.1	3.3	0.3	0.0010^3^

^1^Weighted %

^2^*P* value by chi-squared test

^3^*P* value by *t* test

The food intake results for subjects according to depression are shown in Table 3. Subjects with depression showed a significantly lower intake of total food, legumes and their products, vegetables (including non-salted and salted), fresh fruits, and other food than those without depression in both the unadjusted and adjusted analyses (*P* < 0.05). Intake of seaweeds in the depression group was not significantly lower than that in the non-depression group in the unadjusted results, but the difference became statistically significant after adjustment for sex, age, and energy intake (*P* = 0.0392).

**Table 3:** Food intake of subjects according to depression

	Non-depression (*n* = 4050)		Depression (*n* = 299)		Unadjusted *P* value^1^	Adjusted value^2^
	Mean (g/day)	SE	Mean (g/day)	SE		
Total food	1650.7	18.6	1453.2	65.4	*0.0040*	*0.0016*
Cereals and grain products	295.0	3.4	285.5	12.7	0.4644	0.4818
Potatoes and starches	41.4	2.3	43.0	7.2	0.8220	0.8625
Sugars and sweets	11.3	0.5	11.5	1.9	0.9098	0.7012
Legumes and their products	39.3	1.6	26.8	3.2	*0.0004*	*0.0079*
Seeds and nuts	9.0	0.8	7.6	1.9	0.5212	0.5153
Vegetables	343.6	5.0	291.2	14.5	*0.0005*	*0.0008*
Non-salted vegetables	222.8	4.3	193.0	11.7	*0.0137*	*0.0102*
Salted vegetables^3^	120.8	2.6	98.2	6.6	*0.0011*	*0.0338*
Mushrooms	6.6	0.6	5.2	1.3	0.2868	0.2750
Fruits	200.2	6.0	155.7	16.5	*0.0086*	*0.0005*
Fresh fruits	190.8	6.1	150.6	16.4	*0.0176*	*0.0013*
Fruits preserved in sugar^4^	9.5	1.0	5.1	2.3	0.0763	0.0652
Meat, poultry, and their products	105.3	3.0	89.1	9.8	0.1091	0.5761
Eggs	26.5	1.0	23.4	3.2	0.3388	0.6627
Fish and shellfish	99.3	3.7	82.7	10.8	0.1482	0.2388
Seaweeds	27.0	2.3	16.6	4.9	0.0640	*0.0392*
Milk and dairy products	83.8	3.2	84.1	13.2	0.9871	0.9708
Oil and fats	8.9	0.2	9.2	1.1	0.7819	0.3026
Beverages	312.8	10.9	280.0	29.6	0.3000	0.7325
Seasonings	39.5	1.1	41.3	5.1	0.7185	0.3163
Other food	1.3	0.3	0.4	0.2	*0.0136*	*0.0280*

^1^All *P* values were obtained with the surveyreg procedure in SAS

^2^Adjusted for sex, age, and energy intake

^3^Including vegetable juice, pickles, and kimchi

^4^Including jam and fruit juice

Table 4 presents the intake range, depression, and odds ratios by quartile of non-salted vegetable and fresh fruit intake. According to vegetable and fruit intake quartile, the depression rate of all subjects was 4.7–8.7% and decreased as vegetable and fruit intake increased. Regarding depression ratio by sex, this ratio decreased from 6.4 to 2.5% for males and from 11.4 to 6.6% for females as vegetable and fruit intake increased (sex-related data are not shown). The odds ratios for all, male, and female subjects showed that vegetable and fruit intake was inversely associated with depression with no adjustment (Model 1) (*P* for trend < 0.05). In Model 2, adjusted for age and energy intake, all three groups (all, male, and female) demonstrated a decreasing odds ratio for depression as intake of vegetables and fruits increased (*P* for trend < 0.05). In Model 3 (adjusted for Model 2 + age, energy intake, obesity, smoking, drinking, and stress) and Model 4 (adjusted for Model 3 + eating-out frequency, breakfast, and food security), the total and female groups exhibited significantly lower rates of depression when the intake of vegetables and fruits was high (*P* for trend < 0.05).

**Table 4:** Odds ratio for the presence of depression by fruit and vegetable intake

	Q1 (*n* = 1087)		Q2 (*n* = 1087)		Q3 (*n* = 1088)		Q4 (*n* = 1087)		Total (*n* = 4349)	
	*n*	%^1^	*n*	%	*n*	%	*n*	%	*n*	%
Presence of depression										
Non-depression	985	91.3	1017	94.6	1015	93.1	1033	95.3	4050	93.5
Depression	102	8.7	70	5.4	73	7.0	54	4.7	299	6.5
Fruit and vegetable intake^2^ (g/day)										
Mean, SE	83.2	1.8	246.7	1.8	443.6	2.4	924.5	14.5	409.0	8.0
Median, SE	86.3	3.1	245.5	2.4	437.9	3.5	797.1	12.0	320.4	6.8
Intake range	≦ 160.3		160.5–332.8		332.9–581.5		≧ 582.8		0–3410.6	
	Reference		Odds ratio (95 % confidence interval)					*p* for trend^3^		
Model 1	1		*0.600 (0.419–0.859)*		0.775 (0.544–1.104)		*0.510 (0.353–0.736)*		0.0035	
Model 2	1		*0.577 (0.405–0.822)*		*0.715 (0.513–0.994)*		*0.445 (0.309–0.641)*		0.0002	
Model 3	1		*0.661 (0.437–0.999)*		0.827 (0.538–1.270)		*0.502 (0.340–0.742)*		0.0030	
Model 4	1		0.688 (0.450–1.052)		0.945 (0.612–1.461)		*0.575 (0.385–0.859)*		0.0284	
Model 5	1		0.690 (0.441–1.078)		1.114 (0.720–1.725)		*0.660 (0.438–0.993)*		0.1564	

^1^Weighted %

^2^Only intake of fresh fruit and non-starchy unsalted vegetables

^3^*p* for trend was obtained using the surveylogistic procedure in SAS.

Model 1: Crude

Model 2: Adjusted for sex, age, and energy intake

Model 3: Adjusted for Model 2 + obesity, smoking status, drinking status, stress status

Model 4: Adjusted for Model 3 + average frequency of eating-out per week, breakfast, and food security

Model 5: Adjusted for Model 4 + household income level, area, and marital status

## Discussion

In this study, we used 2014 KNHANES data to examine the correlation between vegetable and fruit intake and depression among Korean adults. We found that higher vegetable and fruit intake was significantly associated with a decreased prevalence of depression. Regarding the relevance of depression according to general characteristics, subjects who were female, aged 30–49 years, unemployed, or with a college or higher education exhibited a higher proportion of depressive symptoms than others. Regarding dietary behavior and prevalence of depression, depression rates were higher among subjects who skipped lunch, were in the “mildly insecure” food security group, ate out 1–3 times/month, or consumed < 400 g of vegetables and fruits per day. Regarding nutrient intake, protein, fiber, calcium, phosphorus, iron, potassium, thiamine, and riboflavin levels were significantly lower in the depression group than in the non-depression group in the unadjusted data. After adjustment for sex, age, and energy intake, only fiber and potassium were significantly lower in the depression group than in the non-depression group. Subjects in the depression group also consumed significantly less seaweed than those in the non-depressed group after adjustment. Significantly, subjects with depression consumed less total food, legumes and their products, vegetables (non-salted and salted), fresh fruits, and other food than those without depression in both unadjusted and adjusted analyses. The odds of depression decreased significantly as the consumption of vegetables and fruits increased among all, male, and female subjects.

Miki et al. [31] investigated the association between dietary fiber and depressive symptoms among 1977 Japanese workers aged 19–69 years. They found that a greater intake of dietary fiber from vegetables and fruits correlated significantly with lower depressive symptoms. Major depression is primarily associated with imbalances in neurotransmitter production and transmission, such as serotonin receptor abnormalities, higher monoamine oxidase (to metabolize serotonin), and abnormalities in the expression of tryptophan hydroxylase (involved in serotonin synthesis) [32–34]. Recent studies have reported that the gut microbiota are important in the gut–brain axis and play a role in modulating brain function by altering the level of cytokines. Dietary fiber from vegetables, fruits, and other plants can help to improve the composition of intestinal microbiota [35].

Our results in this study also indicate that some micronutrients (calcium, iron, thiamin, and riboflavin) were significantly lower in the depression group than in the non-depression group (data not shown). Some essential micronutrients, including calcium, zinc, iron, and folate, play important roles in depression through their regulation of cellular functions and neural transmission [36–40]. The inverse relationship between dietary iron and calcium intake and depression in this study is supported by several epidemiological and meta-analysis studies [40–42]. Calcium and iron are involved in the synthesis of neurotransmitters related to depression, such as serotonin and dopamine [43, 44]. The vitamin B complex, including thiamine and riboflavin, is essential for maintaining healthy immune and nervous systems. Dietary vitamin B deficiency could thus be closely related to mental disorders such as depression, mood disorders, anxiety, and cognitive decline [45]. In a study of 1587 Chinese adults aged 50–70 years, Zhang et al. [46] reported that insufficient thiamine was significantly associated with higher odds of depression. Another study reported that depressive patients who received thiamine supplementation showed improvement in depressive symptoms in as little as 6 weeks [47].

Our findings support previous studies that reported that healthy diets, including high vegetable and fruit intake, reduced the rates of depression and other mental health disorders. McMartin et al. [14] examined the association between fruit and vegetable intake and mental health disorders using a cross-sectional study of Canadians (*n*, 296,121 aged 12 years or older) five times between 2000 and 2009. They found that fruit and vegetable intake was negatively associated with depression, psychological distress, and poor mental health. A meta-analysis of fruit and vegetable consumption and risk of depression (including 227,852 participants for fruit intake and 218,699 participants for vegetable intake) was reported by Lui et al. [48]. They also found that fruit and vegetable intake was inversely related to the risk of depression. The negative association between fruit intake and depression has thus been observed in both cross-sectional and cohort studies.

Johnson et al. [16, 17] reported an association between mental well-being and a community-based healthy living intervention that included greater fruit and vegetable consumption and physical activity. They reported improvements in the mental well-being of participants 3 months after the healthy living intervention. Fruit and vegetable consumption greatly increased over time compared with physical activity, and greater fruit and vegetable consumption was associated with more positive changes in the mental well-being than physical activity. Mihrshahi et al. [15, 16] reported an association between fruit and vegetable intake prevalence and incidence of depressive symptoms in a study of 6271 middle-aged women from the Australian Longitudinal Study on Women’s Health. They found that depressive symptoms were lower among subjects who ate more than two servings of fruits per day and that higher vegetable intake was negatively associated with the prevalence of depressive symptoms.

Kim et al. [49] reported an association between dietary patterns and depression among US adults using two waves (2007–2008 and 2009–2010) of National Health and Nutrition Examination Survey (NHANES) data. They found that the “healthy” dietary pattern (whole grains, vegetables, fruits, fish, nuts and seeds, and oil, with high consumption of protein, dietary fiber, polyunsaturated fat, vitamin C, vitamin A, β-carotene, vitamin E, vitamin D, calcium, and sodium) was negatively related to prevalence of depression in women. On the other hand, the Western dietary pattern did not show any relationship to depression among men or women. Miki et al. [31] examined the relationship between dietary patterns and depressive symptoms in 2006 Japanese employees aged 19–69 years using an empirical dietary pattern method (reduced rank regression). They found that a healthy dietary pattern that included high intakes of vegetables, fruits, mushrooms, seaweeds, soy products, green tea, potatoes, and small fish (including bones) and low rice consumption was negatively associated with depressive symptoms. A cross-sectional study of 2266 Japanese employees aged 21–65 years showed that participants with high scores for the balanced Japanese dietary pattern (high intake of vegetables, including carrots and pumpkin, as well as typical Japanese foods such as mushrooms and seaweed) were significantly less likely than others to show depressive symptoms [4]. Jacka et al. [10, 11] reported that traditional Norwegian and Australian diets that included vegetables, fruit, meat, fish, and whole grains were also associated with a low incidence of depression. Similarly, a study by Sanchez-Villegas et al. [8] demonstrated that the Mediterranean diet might help to reduce depressive symptoms.

This study had some methodological limitations. First, the estimated food intake (including vegetable and fruit consumption) might not accurately reflect subjects’ usual food intake because the survey used the 24-h recall method. Second, the cross-sectional study design means that cause–effect relationships cannot be confirmed between vegetable and fruit intake and depression. For example, the low intake of vegetables and fruits among subjects with depression could be a result of appetite loss, which is a common depressive symptom. Third, our data assessed depression using a self-reported questionnaire (PHQ-9), not medical diagnoses by a specialist.

Despite these limitations, this study also has its strengths. First, it is a population-based study with a relatively high response rate and large sample size. Second, this is the first cross-sectional study to investigate associations between vegetable and fruit consumption and the prevalence of depression in an Asian population. Most research on the association between vegetable and fruit intake and depression has been conducted in European countries. Studies that include Koreans, including our findings, remain very limited. Additional epidemiological and clinical randomized controlled trials are needed to clarify the role of vegetable and fruit intake in depression.

## Data Availability

National data is available by request from the Korean CDC
